# Intelligent Recognition of Sports Players' Wrong Actions in view of Computer Pattern Recognition

This article has been retracted.

**DOI:** 10.1155/2022/5336017

**Published:** 2022-07-04

**Authors:** Rui Guo, Bo Qi

**Affiliations:** ^1^School of Physical Education, Henan University of Technology, Zhengzhou 450001, Henan, China; ^2^Department of Physical Education and Teaching of Central South University, Changsha 410083, Hunan, China

## Abstract

In the context of the vigorous development of the sports industry and rapid technological innovation, the wrong actions of sports athletes can also be intelligently recognized. Human action recognition based on computer pattern recognition is becoming more and more popular and ubiquitous in life. This article aims to study how to recognize the human body based on the computer model and how to apply intelligent recognition to the wrong actions of sports athletes. The study of the application of intelligent recognition to the wrong actions of sports athletes is of great significance to sports athletes. This article proposes how to intelligently recognize the wrong actions of sports athletes based on computer pattern recognition. In the experiment in this article, wrong sports actions can cause a series of undesirable consequences, such as joint sprains and muscle damage. Among them, the proportion of joint damage caused by wrong actions has reached 24% and has been rising with the increase of the number of experiments and finally reached 35%, which shows that the probability is still very high. After the pull-up adopts intelligent recognition, the error of the pull-up action can be quickly identified and corrected in time, with the correct rate reaching 78%. Therefore, in order to reduce the physical damage caused by sports athletes' wrong movements, it is necessary to study the intelligent recognition of sports athletes' wrong movements. The recognition of wrong actions of sports athletes can be carried out through intelligent recognition based on 3D convolutional neural networks, which is of great significance to intelligent recognition.

## 1. Introduction

With the development of computer technology and the progress of society, more and more jobs are replaced by computers. In recent years, due to the great progress of computer vision technology, computers have replaced many applications and completed more and more tasks. However, letting computers think like humans and understand the world like humans is a big problem. Therefore, many scholars are concentrating on the computer field [1, 2]. In order to enable computers to judge and recognize external information autonomously, they are studying ways to make computers smarter.

In the field of computer vision, the recognition of human action is always an active topic. Among them, the method based on video sequence is widely used in the recognition of human action. Research content on human motion analysis based on video sequences mainly includes computer vision systems, computer graphics, image processing, image recognition, artificial intelligence, and other fields. This is an academically challenging research topic. The research methods of human action recognition include digital image processing, image recognition, artificial intelligence, and other fields. Sports is based on the laws of human anatomy and physiology and is composed of a series of movements. The correctness of these actions is directly related to whether they can effectively enhance physical fitness and create sports performance. Only by following the laws of sports and ensuring that the movements are accurate can the potential be released and the value of sports can be truly brought into play. Therefore, athletes must discover and correct their wrong actions in time. The wrong actions of sports players based on computer pattern recognition can improve the correct rate of athletes' actions and prevent athletes from being injured. The research on this subject has very important practical significance and application value.

With the development of sports in recent years, the importance of intelligent recognition has become higher and higher. Uddin and Kim found that human activity recognition based on computer vision has become very famous because of its applications in various fields such as smart home medical treatment. Video-based activity recognition systems basically have many goals, such as responding to people's behavior so that the system can actively assist them in completing tasks. In their work, they proposed a new method of deep body shape and deep learning network. Finally, these features are used to train a deep learning network for later recognition. The HAR method they proposed shows better performance than traditional methods on private and public datasets, which shows that it is an outstanding method for practical applications in intelligent control environments [3]. Kamal found that human behavior assessment during routine operations in indoor areas plays an important role in healthcare services. During this consideration, a depth camera is initially used to capture depth images and segment human contours due to color and intensity changes. The features consider the temporal and spatial characteristics and are obtained from the human body color joints and depth contour information. By obtaining joint displacement and specific motion characteristics from human color joints and processing the side frame distinguishing characteristics according to the depth data, the classification performance is improved [4]. Santhoshkumar and Geetha found that analyzing human movement for emotion recognition is essential for social communication. Nonverbal communication methods such as body movements, facial expressions, gestures, and eye movements are used in a variety of applications. Among them, the advantage of emotion recognition through body movements is that it can recognize the emotions of people from any camera perspective. Compared with other studies, physical exercise can strongly convey emotional states. They used a feedforward deep convolutional neural network architecture with different parameters to recognize emotional states from whole body motion patterns. Experimental results show that the system has good recognition accuracy [5]. Wang et al.'s research puts forward a new radar-based recognition method of human body and limb movement, which takes advantage of the temporal sequence of movement. A stacked gated recurrent unit network (SGRUN) is used to extract dynamic sequential human motion patterns. Since time-varying Doppler and micro-Doppler features can well represent this movement pattern, the spectrogram is used as the input sequence of SGRUN. Numerical experiments verify that SGRUN with two 34-neuron-gated cyclic unit layers can classify and recognize six different types of human and limb movements [6]. Li et al. found that body posture is an important indicator of human behavior. Existing gesture-based action recognition methods are usually designed for a single human body and require a fixed size, such as an input vector. They proposed a method of deep neural network architecture. To this end, they designed a human pose coding scheme to eliminate the requirements and provide a general representation of two-dimensional human joints, which can be used as the input of CNN. In addition, they also proposed a weighted fusion scheme. Evaluating the method on two real-world datasets, compared with the most advanced methods, their method has achieved better performance [7]. Shao et al. found that people are paying more and more attention to identifying human movements from skeletal data. By proposing a hierarchical model to discover the structural information of the body parts involved in the action, they can better analyze the human actions in the skeleton data, so as to focus on such tasks. Regarding human behavior as the simultaneous movement of human bones and body parts, they proposed a layered model. It simultaneously applies the discriminative body part selection of the same scale and the group coupling of body part bundles of different scales. It decomposes the human skeleton into a hierarchical structure of body parts of different scales [8]. Li et al. found that Human Activity Recognition (HAR) in wearable devices is a promising technology in pervasive computing. However, traditional methods often regard human activity recognition as a single tag recognition problem, ignoring the correlation between current activity patterns, personal movement patterns, and sensor wearing positions. They proposed a multitask human activity recognition multitask learning framework based on supervised learning. They extract the time domain and frequency domain features of the original data and classify the data through a multitask learning framework composed of a fully connected network and a convolutional neural network, which can achieve high accuracy [9]. Zhang et al. proposed a new human activity recognition technology based on deep learning. They used convolutional neural networks (CNN) to extract features from BSTM and classify activities. In order to evaluate this method, they conducted several tests, and the experimental results show that the technology is superior to the traditional state-of-the-art methods in recognition accuracy and provides performance comparable to recent deep learning techniques [10]. Through the experimental analysis of scholars, it can be known that intelligent human body action recognition is used more and more widely, and it is more and more recognized by people, so intelligent recognition can also be well applied to sports actions. The analysis of scholars emphasized the advantages of intelligent recognition, but the experimental data were neglected. Too little data reduce the authenticity of the experiment.

The innovations of this article are as follows: (1) the theoretical knowledge of computer pattern recognition and sports athletes' wrong actions is introduced, and the body movement recognition algorithm is used to analyze how intelligent recognition affects sports athletes' wrong actions for research; (2) this article conducts experimental analysis on the 3D convolutional neural network algorithm and conducts experiments and analysis on the movement of students in physical education colleges. Through experiments, it is found that intelligent recognition can effectively correct the wrong actions of sports athletes and improve the accuracy of the actions.

## 2. Human Action Recognition Algorithm Based on Computer Recognition

In recent years, computer vision characteristic analysis and image processing technology have been widely used for the analysis of various shapes and structures of the moving human body by computer image processing technology [11, 12]. The human body recognition algorithm uses big data and deep learning technology to detect the human body from images and videos, recognize the human body's behavior, and track the characteristics of the human body. It helps machines and smart products recognize whether there is a human body passing by and recognize different human postures and body movements. Also, it can walk with the human body, which can be applied in many fields. At the same time, in the field of sports, in order to improve the effectiveness and judgment of athletes' training, computer vision characteristic analysis technology has been introduced into the recognition and correction of athletes' actions [13]. Computer vision technology mainly uses visual feature extraction methods to recognize the effective actions of athletes when performing athlete action recognition and evaluate the accuracy of the actions accordingly. In the understanding of athletes' improper behavior, the 3D visual inspection modeling method is mainly used to form the 3D visual discriminant function of athletes' improper behavior and construct the 3D visual detection model of improper behavior. Then, the athlete evaluates the wrong behavior during the exercise. Intelligent recognition is related to the development of the sports industry and has attracted the attention of people in the industry, and certain results have been achieved in some studies [14]. Intelligent recognition in motion is shown in Figure 1.

As shown in Figure 1, with the rapid development of sensor technology, the maturity of the Internet, and mechanical learning theory, human action recognition technology has attracted more and more attention from researchers [15, 16]. Human-machine motion recognition technology has high academic and commercial value and is suitable for various scenarios such as human-computer interaction, intelligent surveillance, dynamic analysis, and video retrieval. The effect of traditional human behavior recognition methods largely depends on the advantages and disadvantages of manually extracted features [17]. The calculation process of features is complicated, and the generalization of extracted features is not strong. This paper uses deep neural network to simulate the visual information processing process of the biological brain and realizes the feature extraction of human motion in the video. It can adapt to human behavior recognition in complex environments, simplify the process of traditional artificial features, and improve recognition accuracy [18–20].

### 2.1. Human Action Recognition Algorithm Based on Time-Frequency Features

Time-frequency distribution is a tool that allows people to observe the time domain and frequency domain information of a signal at the same time, and time-frequency analysis is to analyze the time-frequency distribution. Traditionally, Fourier transform is used to observe the frequency spectrum of a signal. Human body motion is a kind of nonlinear motion, and the commonly used linear dimensionality reduction methods cannot effectively extract the key information in the action characteristics. The content of this chapter starts with the time-frequency characteristics of motion capture data and realizes the recognition of human actions by introducing a new nonlinear dimensionality reduction method to reduce the dimensionality of the action features [21]. Compared with the linear dimensionality reduction method, this method greatly improves the accuracy of action recognition.

In the past many years, both microelectronics and computer systems have achieved rapid development and multiple sensors and mobile terminals with special performance have continued to appear. Because of the emergence of these high-performance, portable, and low-power smart devices, the method of interaction between humans and computers has undergone great changes. People are no longer satisfied with traditional information dialogue methods such as mouse and keyboard, but need more convenient and faster dialogue methods that can adapt to humans and computers [22]. As a method of interaction between the external environment and spontaneous information, the movement of the human body contains important information such as body language and emotional color.

In order to realize the real-time recognition of human movements, it is necessary to window the motion capture data, that is, to divide the data into a short sequence of specified length. At the same time, in order to enhance the ability to describe actions, there is a 50% overlap between adjacent windows [23]. The length of the window is related to the frequency of human behavior. If the length of the window is shorter, the cycle of human body movement included is also less and the recognition effect is also worse. If the length of the window is longer, the cycle of human body movement included is more and the recognition effect is more stable. After data segmentation of the action sequence, the characteristics of each dimension signal in the window in the time domain and frequency domain are extracted. The calculation of time domain features is relatively simple, as shown in the following equation:

(1) $$\begin{array}{c} \sigma^{2}=\frac{1}{M}\sum_{M-1}^{M}\left(a_{i}-\mu_{i}\right), \end{array}$$

where *M* represents the segmentation length of the action sequence and *μ*_*i*_ represents the value of the *i*-th dimension feature in the feature vector at the *M*-th moment.

After the signal is transformed by FFT, the frequency domain characteristic *H* of the signal is extracted, as in the following equation:

(2) $$\begin{array}{c} H=-\sum_{K=1}^{M}a_{i}k\;\log_{2}a_{i}\left(k\right). \end{array}$$

In order to eliminate the influence of the dimension and value range of the features of different dimensions in the feature vector, this paper uses formula (1) to normalize the features of different dimensions. Map the features of each dimension to the range of [0,1], as in the following formula:

(3) $$\begin{array}{c} b_{i}=\frac{a_{i}-\min\left(f_{i}\right)}{\max\left(f_{i}\right)-\min\left(f_{i}\right)}, \end{array}$$

where min(*f*_*i*_) and max(*f*_*i*_) are the minimum and maximum values of the *i*-th dimension feature, respectively, and *a*_*i*_ is the value of the *i*-th dimension feature.

At present, the dimensionality reduction methods applied to action features are mainly traditional linear dimensionality reduction methods. The two methods of this method are linear discriminant analysis and principal component analysis. However, this type of method cannot extract the important information from the action features well. Generalized discriminant analysis is a nonlinear dimensionality reduction method that is rarely used in the field of human action recognition [24]. This article focuses on the introduction of linear discriminant analysis. Linear discriminant analysis is a generalization of linear discriminant methods. This method uses statistics, pattern recognition, and machine learning methods to try to find a linear combination of the characteristics of two types of objects or events to be able to characterize or distinguish them.

Suppose the action feature matrix *A*=(*a*_1_, *a*_2_,…, *a*_*n*_), where *Q* is the number of action samples and *a*_*n*_ is the feature vector corresponding to the *i*-th action sample. These feature vectors belong to *C* different action categories. The intraclass divergence *Q*_*W*_ of the action feature vector is expressed as follows:

(4) $$\begin{array}{c} Q_{W}=\sum_{I=1}^{C}\left(\mu_{i}-a_{i}\right){\left(\mu_{i}-a_{i}\right)}^{T}. \end{array}$$

Among them, *μ*_*i*_ represents the average value of all feature vectors in the *i*-th action category and (*μ*_*i*_ − *a*_*i*_)^*T*^ represents the average value of all feature vectors.

According to the definition of linear discriminant analysis, the goal of linear discriminant analysis is to obtain the maximum value of formula (4) by solving the projection vector W, as in the following equation:

(5) $$\begin{array}{c} J\left(W\right)=\frac{\left|W^{T}Q_{B}W\right|}{\left|W^{T}Q_{W}W\right|}. \end{array}$$

Since the multiple change of *W* will not change the solution goal *J*(*W*), the denominator is simplified to 1, which is |*W*^*T*^*Q*_*W*_*W*|=1. Therefore, the *J*(*W*) maximization problem is transformed into the following optimization problem with constraints, such as

(6) $$\begin{array}{c} \min W=-\frac{1}{2}W^{T}Q_{B}W. \end{array}$$

KKT condition is a very important concept and method in solving optimization problems with inequality constraints. According to the KKT condition, the solution of formula (5) is the same as that of formula (6). Therefore, the original problem is transformed into the problem of solving the eigenvector corresponding to the larger eigenvalue after eigenvalue decomposition of min*W* [25].

After the dimensionality of the action feature is reduced, the feature vector corresponding to several eigenvalues will be discarded. This approach has two advantages: first, by discarding part of the information, the samples of the same kind can be clustered closer together, thereby increasing the density of the samples. Second, a small amount of noise is often introduced in the sample collection process and part of the noise can be effectively removed by discarding part of the information [26].

### 2.2. Algorithm of Support Vector Machine

Support vector machine is a kind of generalized linear classifier that classifies binary data in a supervised learning manner, and its decision boundary is the maximum margin hyperplane for solving learning samples. After modeling the human body, in order to describe the actions of the human body, some features of the human body model in each frame of the image are selected, such as the trajectory and speed of the hand movement when the person is waving. At the same time, it has information on the physical movement of the elbow joints involved in the hand [27]. The joints of the human body have high degree of freedom and complex movements. If a movement is described by the feature information of all joints, each feature is a dimension, and the total number of dimensions of the movement data will be very large. This is called a dimensional disaster. In machine learning, this type of data is prone to overfitting [28]. Considering the time cost and performance of the algorithm, it is necessary to perform feature selection on the original data. The process is shown in Figure 2.

As shown in Figure 2, it uses this part of features with high degree of distinction and good uniformity to form a feature subspace. The feature transformation is to map the original feature space to the low-dimensional feature space according to the method.

With its excellent performance, support vector machines have received extensive attention and recognition in the field of pattern recognition and machine learning in recent years. It shows not only a higher accuracy rate in classification problems but also a higher generalization ability. Many authorities even think it is the best. Therefore, support vector machines are also widely used. Support vector machine is a discriminative classification method, but it is different from many learning methods. The difference is that other algorithms generally use all samples for training and then use gradient descent, least squares, and other algorithms to iterate until the result of the operation converges, and the corresponding classification algorithm model can be obtained [29].

The principle of support vector machine is to determine the classification hyperplane of the sample space by only relying on the distribution of some samples. The part of the feature that determines the classification hyperplane is the so-called support vector. Therefore, during training, the part of the data far away from the classification hyperplane does not contribute to the classification model. The classification hyperplane determined by the support vector realizes the linear separability of the entire sample space. The distance to the support vector is the largest, and it has a good classification ability for unknown data [30]. The support vector machine is shown in Figure 3.

As shown in Figure 3, support vector machine training refers to the calculation of sample data to determine the classification hyperplane with the largest distance. The maximum distance here is the maximum distance of the geometric interval, and it is also the minimum distance to the hyperplane in all the training data. The following is the definition of the classification discriminant function:

(7) $$\begin{array}{c} \gamma^{i}=b_{i}\left({\left(\frac{\omega }{\left\|\omega \right\|}\right)}^{T}+\left(\frac{b}{\left\|\omega \right\|}\right)\right). \end{array}$$

Among them, (*ω*, *b*) is the parameter of the classification hyperplane. If the sample falls on the classification hyperplane, then formula (8) is satisfied:

(8) $$\begin{array}{c} \omega^{T}a+b=0. \end{array}$$

The parameter *ω*=[*θ*_1_,…,*θ*_*n*_]^*T*^ of the hyperplane needs to be determined by training. The calculation idea is to transform the parameter solving problem into a convex quadratic programming solvable optimization problem:

(9) $$\begin{array}{c} \min_{\gamma ,\omega ,b}=\frac{1}{2}{\left\|\omega \right\|}^{2}. \end{array}$$

For formula (9), Lagrangian dual transformation is introduced in the calculation. A kernel function is introduced in the transformation, and the kernel function maps high-dimensional linearly inseparable samples to low-dimensional linearly separable samples. Bringing the kernel function into the decision function has

(10) $$\begin{array}{c} f\left(a\right)=\sum_{i=1}^{n}\alpha_{i}b_{i}k\left(a,a_{i}\right)+b, \end{array}$$

where *n* represents the number of support vectors, *α* is the Lagrangian multiplier, each sample corresponds to a Lagrangian multiplier, *b* represents the offset of the classification hyperplane, *K* is the kernel function, and *b*_*i*_ are *a*_*i*_ and are generally classified as 1 or −1.

Convolutional neural network imitates the construction of biological visual perception mechanism, which can perform supervised learning and unsupervised learning. The convolution kernel parameter sharing in the hidden layer and the sparsity of the connections between layers enable the convolutional neural network to lattice features with a small amount of calculation, for example, pixel and audio learning, stable effects, and no additional feature engineering on the data, as shown in Figure 4.

As shown in Figure 4, among them, the simple and regularized image is input into the network through the input layer, and through the local receptive field, the neurons in each layer are connected with a group of local neighbor neurons in the previous layer. The local receptive field can extract some basic visual features such as directed edges and end points [31]. A convolution kernel sliding on the image acquires a feature of the image and forms a feature map.

#### 2.2.1. Convolutional Layer

The result of the operation is as follows:

(11) $$\begin{array}{c} b_{mm}=f\left(\sum_{j=0}^{j-1}\sum_{j=0}^{j-1}a_{m+1,n+1}w_{ij}+b\right). \end{array}$$

Among them, *a* is the input image matrix, 2 is the weight matrix of the convolution kernel of size *J* × *I*, *b* is the bias and the output value of *M* × *N*, and *b*_*mm*_ is the activation function.

#### 2.2.2. Average Pooling Layer

The average pooling layer calculates the average value of all points in a sampling window as the sampling result. The calculation process is as follows:

(12) $$\begin{array}{c} b_{mm}=\max\left(a_{m\times s_{i}}+b_{m\times s_{i}}\right). \end{array}$$

Among them, *a* is the two-dimensional input matrix, *b* is the output obtained after sampling, and *m* and *s* are the positions of the target pixels. *S*_1_ and *S*_2_ have the sampling step length in the horizontal and vertical directions, respectively, which stipulates the size of the sampling window. In the downsampling stage, most of the window nonoverlapping strategies are adopted, that is, each sampling window is connected and does not overlap. Downsampling can quickly reduce the data size and reduce the amount of network calculations [32].

#### 2.2.3. 3D Convolution

When building a 3D convolutional neural network model, various convolution kernels need to be used to extract various features. In the direction from input to output, the number of feature cubes gradually increases, so as to generate more cube-combined type characteristics from lower features. The convolution kernel of the neural network is a three-dimensional cube. In the network, each feature cube of the convolutional layer can be connected to multiple adjacent continuous frames of the previous layer to capture motion information within a certain period of time [33, 34]. The three-dimensional convolution process is shown in Figure 5.

As shown in Figure 5, the same 3D convolution kernel shares weights and offsets in the entire frame cube, so a convolution kernel can only extract one type of feature.

The position of the *m*-th feature cube in the *l*-th hidden layer and the output value of the neuron at *b*_*lm*_ are calculated as follows:

(13) $$\begin{array}{c} b_{lm}^{ijk}=f\left(b_{lm}+\sum \sum_{p=0}^{p_{l}-1}\sum_{q=0}^{q_{1}-1}\sum_{R=0}^{RI-1}w_{lmn}^{pqr}a_{\left(l-1\right)n}^{\left(i+p\right)\left(j+q\right)\left(k+r\right)}\right), \end{array}$$

where *b* is the output at (*l*, *j*, *k*) of the *l*-th layer, *a* is the input from the *i*-th hidden layer to the *l-*th layer, the size of the l-th layer convolution kernel is *P* × *Q* × *R*, and *f*(*A*) is the activation function. *b*_*lm*_ is the offset shared by the feature cube, and *n* is the index of the feature cube connected to the current feature cube at layer *l−*1. *w*_*lmn*_^*pqr*^ is the weight between the neuron at the location (*p*, *q*, *r*) of the *m*-th feature map of the *l*-th layer and the *n*-th feature map of the *l−*1 layer.

The three-dimensional maximum pooling formula is as follows:

(14) $$\begin{array}{c} b_{i,j,k}=\max\left(a_{i}\times s_{i}\right). \end{array}$$

Among them, *s*_*i*_ is the sampling step. After sampling, the size of the feature map is reduced and the amount of calculation is greatly reduced.

This paper introduces the frame difference channel based on visual attention in the input layer of the 3D convolutional neural network and expands the input of the constructed neural network model to dual channels. It inputs the frame difference matrix as another channel into the neural network model along with the original gray-scale video frame cube.

Among them, the frame difference channel uses the three-frame difference method for calculation. By taking the adjacent three frames of images as a group for redifferentiation, it can better detect the before and after changes of the intermediate frame. The three-frame difference algorithm is an improved method of the adjacent two-frame difference algorithm. It selects three consecutive frames of video images for differential operation, eliminates the influence of the exposed background due to motion, and extracts accurate contour information of the moving target. The frame difference can describe the difference of human body movement during the movement, and the area that should be paid attention to in the whole frame cube is described by the frame difference matrix.

Select two consecutive frames of images *I*_*t*_(*a*, *b*) and *I*_*t*−1_(*a*, *b*) in the video frame sequence to calculate the difference between two adjacent frames as follows:

(15) $$\begin{array}{c} D_{t,t-1}\left(a,b\right)=\left|I_{t}\left(a,b\right)-I_{t-1}\left(a,b\right)\right|. \end{array}$$

For the obtained difference image, the insignificant change area is proposed by selecting the appropriate threshold *T* and the noise interference is eliminated as follows:

(16) $$\begin{array}{c} W\left(a,b\right)=\left\{\begin{array}{c} D_{i}\left(a,b\right),D_{I}\left(a,b\right)\geq T,\\ 0,D_{i}\left(a,b\right)\geq T. \end{array}\right.. \end{array}$$

In one group, two differential image logics will be obtained and the union of the change areas between two consecutive frames will be obtained. The before and after significant change areas *W*(*a*, *b*) of the intermediate frames in the three frames of images will be obtained as follows:

(17) $$\begin{array}{c} W\left(a,b\right)=\max\left(W_{1}\left(a,b\right),W_{2}\left(a,b\right)\right). \end{array}$$

Finally, the obtained difference image is normalized and the frame difference *Q*(*a*, *b*) is obtained. This three-dimensional matrix can represent the significant change area of the action in the input human behavior video, which is

(18) $$\begin{array}{c} Q\left(a,b\right)=\frac{Q\left(a,b\right)-\min a_{1}}{\max a_{1}-\min a_{1}}. \end{array}$$

If the activation function is used in the output layer, the log-likelihood cost function is used. The formula of the log-likelihood cost function is

(19) $$\begin{array}{c} C=-\sum_{k}b_{k}\log\;a_{k}. \end{array}$$

Among them, *a*_*k*_ represents the output value of the *k*-th neuron and *b*_*k*_ represents the true value corresponding to the *k*-th neuron, with a value of 0 or 1.

In general, the method proposed in this chapter has a good performance on the human body movement dataset collected in a simple environment. The model can be applied to the fields of intelligent monitoring and motion analysis in fixed scenes and has good portability.

## 3. Experiment and Analysis Based on Questionnaire Survey and Convolutional Neural Network Algorithm

### 3.1. Experiment and Analysis of Questionnaire Survey

When athletes conduct sports training, the correctness of the movements is not only related to the practice joints at this stage but also has a certain impact on the athletes before and after the sports training. For example, when practicing high jump, if the body of an athlete who is in the approaching stage depicting the arc of the high jump jumps early, the balance will collapse and the athlete will fall onto the crossbar before jumping.

With the continuous development of information technology, the emergence of computers with stronger computing capabilities and more accurate sensors has also promoted the development of mankind. New technology words such as cloud computing, big data, Internet of Things, and artificial intelligence quickly rushed into various fields and disciplines of various industries and brought changes. At the same time, a more natural and harmonious human-computer interaction mode is also desired by the world.

This article surveys 10 male and 10 female athletes. The experiment allowed them to exercise several times a day. By observing the difference between before and after they use smart recognition, the basic situation of the survey subjects is shown in Table 1.

As shown in Table 1, the age of the survey subjects is generally around 20 years, the interval is 18–23 years, and the number of exercises of the survey subjects is around 15–25 times.

This article investigates and analyzes the consequences of wrong actions in sports, as shown in Figure 6.

As shown in Figure 6, posture errors during exercise belong to actions that do not comply with the requirements of human anatomy during exercise. Do not follow the requirements of human anatomy; the wrong posture may cause joint sprains, muscle tension, and severely tense muscles and tendons. Wrong exercise posture may damage the spine, and severe cases may cause persistent back bends. Among them, the probability of joint sprains was the largest, increasing from 24% to 35%; muscle injuries ranked second, increasing from 16% to 19%.

In sports, in the process of learning various sports skills and learning, there are bound to be various wrong behaviors. If the wrong behavior is not corrected within time, students will develop the habit of wrong behavior. This seriously affects the physical health and training progress of the students. Experiments must not only correctly master the technology and skills but also improve the students' physical fitness and prevent accidents that may occur. Therefore, this article analyzes the benefits of intelligent recognition of wrong actions to students.

In order to verify the function of intelligent recognition, this article compares the correctness of the action before and after running warm-up before and after using intelligent recognition, as shown in Figure 7.

Analyzing Figure 7, we can see that, with the continuous increase of the number of experiments, when the action before warm-up is not intelligently recognized, the accuracy of the action is only about 30% on average. Not only can athletes fail to detect whether their actions are correct, but they may also cause physical damage. Also, after taking the action of intelligent recognition and correcting, the accuracy rate reached about 80% on average. The correct rate of the action before the running warm-up before intelligent recognition is very low. The athletes themselves cannot find out if their actions are wrong. After adopting intelligent recognition, although their actions are wrong, they can be quickly corrected, thereby improving the correct rate of sports athletes' movements.

In order to increase the reliability of the experiment, this article has performed a statistical comparison of the accuracy and recognition rate of several other sports actions before and after using intelligent recognition, as shown in Tables 2 and 3.

As shown in Table 2, this article mainly conducts experiments on pull-ups, squats, standing long jumps, and jumps in sports. The accuracy of pull-ups before intelligent recognition is 78%, and the correct rate is 56%. It can be seen that sports actions that do not use intelligent recognition are prone to errors.

As shown in Table 3, this article mainly conducts experiments on pull-ups, squats, standing long jumps, and jumping in sports. The accuracy of pull-ups after using intelligent recognition is 94%, and the correct rate is 95%. It can be seen that the sports action using intelligent recognition is very standardized. The test results show that the recognition rate of motion recognition is very high and the motion recognition function is very reliable.

### 3.2. Experiment and Analysis of Convolutional Neural Network

In convolutional neural networks, choosing the size of the convolution kernel has a great impact on network performance and classification accuracy. The large-size convolution kernel brings a larger acceptance range and can extract richer features. However, it means that more parameters and more calculations are required. The experimental results of different sizes of convolution kernels in the network construction process are shown in Table 4.

As shown in Table 4, the time required for a forward calculation of a smaller product core is only 0.0093. As the size of the convolution kernel increases, it takes longer. The convolution kernel using 6 × 6 × 6 can achieve the highest classification accuracy rate of 94%. The classification accuracy of the convolution kernel using 4 × 4 × 4 is 93%. The classification accuracy of the convolution kernel using 8 × 8 × 8 is 89%, which is the lowest.

In order to verify the accuracy of the convolutional network intelligent recognition application, this paper analyzes through the comparison of two experiments, as shown in Figure 8.

It can be seen from Figure 8 that the convergence speed of the convolution kernel using 4 × 4 × 4 is faster and the classification accuracy is only slightly lower than that of the 6 × 6 × 6 convolution kernel. However, the use of a 8 × 8 × 8 size convolution kernel has low recognition accuracy and time-consuming calculations. In general, the best network classification performance can be obtained by using a 4 × 4 × 4 size convolution kernel.

The improved dual-channel 3D convolutional neural network is used to identify the wrong behavior of the movement. Using a 3D convolutional neural network, after simple preprocessing, it can directly use the data as the network input. Compared with the method of manually extracting traditional action features, it can avoid the complex feature extraction and data reconstruction process of traditional action recognition algorithms. The original video data information is used to capture deep features. Compared with the 2D convolutional neural network, the 3D convolution kernel can also perform feature extraction in the time dimension. It enables the network itself to learn the characteristics of the time dimension and make sports. Compared with the previous 3D convolutional neural network, the attention mechanism is introduced. By inputting the interframe difference result as another channel into the network, it gives higher attention to the significant difference area of the moving human body and better extracts the characteristics of different behaviors.

## 4. Discussion

Based on computer pattern recognition, this paper explores the method of intelligent recognition of wrong actions of sports athletes to improve the wrong actions in sports. It studies related theories such as the intelligent recognition of wrong actions by sports athletes and discusses whether intelligent recognition can reduce the error rate of wrong actions through experiments.

This paper also makes reasonable use of the support vector machine algorithm based on computer mode, the human action recognition algorithm based on time-frequency features, and the convolutional neural network method based on deep learning. As the combined application range of these algorithms has become larger and larger, their importance has also increased. According to the calculation, it is very meaningful to analyze the intelligent recognition of sports athletes' wrong actions based on computer pattern recognition.

Through the experiment of intelligent recognition of sports athletes' wrong actions, this article shows that the probability of wrong actions in sports is increasing and the impact of wrong actions is very bad. It not only makes sports impossible to complete but also damages the athlete's body. Therefore, it is indispensable to intelligently recognize and correct wrong actions in sports based on computer recognition.

## 5. Conclusion

The focus of this article is to describe the intelligent recognition of sports athletes' wrong actions based on computer pattern recognition. This article gives a detailed introduction to the development of computers and its importance and proposes some algorithms based on computers, e.g., support vector machine algorithms and human action recognition algorithms based on time-frequency features. Among them, this article focuses on the convolutional neural network algorithm. According to the article, 3D convolutional neural network can play a very good effect on human action recognition and the accuracy rate is also very high. Therefore, in the same way, the 3D convolutional neural network can be applied to the intelligent recognition of wrong actions in sports. In the experiment part, a number of students in physical education colleges were investigated and men and women were subjected to experimental analysis of daily exercise movements. Through investigations, it was found that if the athlete's actions are wrong, it will cause many undesirable consequences, such as muscle damage, poor sleep quality, and spine problems. Moreover, there are many wrong actions without intelligent recognition and the accuracy of actions is very low. However, the accuracy of the action using 3D convolutional neural network intelligent recognition is much higher. On the basis of reducing the action error rate, it reduces the risk of athletes being injured. Therefore, research on the intelligent recognition of wrong actions in sports is of great significance.

## Figures and Tables

**Figure 1:** Smart recognition in sports.

**Figure 2:** Feature selection process.

**Figure 3:** Schematic diagram of support vector machine.

**Figure 4:** Convolutional neural network.

**Figure 5:** Three-dimensional convolution process.

**Figure 6:** The consequences of wrong actions in sports.

**Figure 7:** Correct rate of action before and after running warm-up before and after smart recognition. (a) Action accuracy rate before running warm-up before intelligent recognition. (b) Action accuracy rate before running warm-up after intelligent recognition.

**Figure 8:** The accuracy of different sizes of convolutional networks in intelligent recognition applications. (a) The accuracy rate of the first convolutional network of different sizes. (b) The accuracy rate of the second convolutional network of different sizes.

**Table 1:** Basic information of the survey subjects.

Survey object	Age	Number of exercises
1	21	16
2	23	15
3	20	17
4	18	15
5	19	15
6	20	19
7	21	20
8	22	25
9	20	20
10	19	25

**Table 2:** Accuracy and recognition rate before using intelligent recognition.

Sport category	Number of exercises	Motion recognition rate (%)	Accuracy (%)
Squat	100	78	56
Pull-ups	150	57	60
Long jump	140	50	65
Jump	160	49	50

**Table 3:** Accuracy and recognition rate after using smart recognition.

Sport category	Number of exercises	Motion recognition rate (%)	Accuracy (%)
Squat	100	90	97
Pull-ups	150	94	95
Long jump	140	95	96
Jump	160	90	92

**Table 4:** Experimental results of convolution kernels of different sizes.

Convolution kernel size	Correct rate (%)	Time-consuming forward calculation (S)
4 × 4 × 4	93	0.0093
6 × 6 × 6	94	0.0032
8 × 8 × 8	89	0.0652

## Data Availability

The data that support the findings of this study are available from the corresponding author upon reasonable request.
